RETRACTED

# Gut Microbiota Variations between Henoch-Schonlein Purpura and Henoch-Schonlein Purpura Nephritis

**DOI:** 10.1155/2022/4003491

**Published:** 2022-04-14

**Authors:** Fang Zhou, Qimin Shao, Lihong Jia, Chunyan Cai

**Affiliations:** Department of Rheumatoid Immune Nephrology, Hangzhou Children's Hospital, Hangzhou, 310014 Zhejiang, China

## Abstract

**Background:**

In China, little is known regarding the differences between children with Henoch-Schonlein purpura (HSP) and Henoch-Schonlein purpura nephritis (HSPN) concerning their gut microbiota.

**Methods:**

We recruited 25 children with HSP, 25 children with HSPN, and 25 healthy children to investigate the differences. Fecal samples were collected and analyzed by sequencing the V3-V4 region of the *16S rRNA* gene. The diversity of the fecal gut microbiota was compared between the patient groups.

**Results:**

Rarefaction curves showed that the gut microbial diversity between the three groups differed significantly (*P* = 0.0224). The top five most abundant gut microbial genera were *Bacteroides*, *Faecalibacterium*, *Prevotella*, *Ruminococcaceae*, and *Megamonas* in children with HSP; *Bacteroides*, *Faecalibacterium*, *Prevotella*, *Bifidobacterium*, and *Ruminococcaceae* in children with HSPN; and *Bacteroides*, *Prevotella*, *Faecalibacterium*, *Ruminococcaceae*, and *Bifidobacterium* in healthy children. Children with HSP had the lowest *Bifidobacterium* abundance among the three groups (*P* < 0.05). Children with HSPN had a lower abundance of *Akkermansia* than children with HSP (*P* < 0.05), whereas children with HSPN had a higher *Alistipes* abundance than children with HSP (*P* < 0.05). Fecal microbial community composition did not differ significantly between groups (ANOSIM, *R* = −0.002, *P* = 0.46). Despite the small sample size, our results indicate that children with HSP or HSPN displayed dysbiosis of the gut microbiota.

**Conclusion:**

This study provides valuable insights that will benefit the development of future microbe-based therapies to improve clinical outcomes or prevent the incidence of HSP or HSPN in children.

## 1. Introduction

Henoch-Schonlein purpura (HSP) is the most common vascular allergic hemorrhagic disease that occurs during childhood [1, 2], affecting 10–20 children per 1,000,000 children, with a peak incidence between 4 and 6 years of age. Primary clinical characteristics include nonthrombocytopenic purpura, arthralgia, abdominal pain, and renal involvement [3]. Long-term prognosis is heavily dependent on the degree of kidney failure. In HSP patients, the microbiome diversity and richness were shown to be reduced. The microbiota composition of HSP patients differed from that of healthy controls. Clinical indicators were linked to the gut microbiota. Henoch-Schonlein purpura nephritis (HSPN) occurs in approximately 30% to 50% of the patients diagnosed with HSP [4, 5]. In these patients, the risk of kidney failure ranges from 2% [6] to 20% in specialized centers [7, 8]. Patients with HSPN present with diverse clinical manifestations, including microalbuminuria to massive proteinuria, microscopic hematuria or hematuria, nephrotic syndrome, acute renal insufficiency, and acute rapidly progressive glomerulonephritis [9]. In HSPN patients, the gut microbiome community richness and diversity were reduced, and the gut microbiota structure was clearly distinct. In HSPN patients, a genus-level comparison revealed a significant increase in the proportions of g-Bacteroides, g-Escherichia–Shigella, and g-Streptococcus, as well as a significant decrease in g-Prevotella 9, implying that the dysbiosis was characterized by an overrepresentation of potential pathogens and a reduction of profitable strains. Although the etiology of HSP remains unknown, available evidence indicates that both genetic and environmental factors are involved, with genetic polymorphisms playing an important role in the development of HSP and the determination of clinical characteristics [10, 11]. Some studies suggest that HSP and HSPN are systemic inflammatory diseases caused by a dysfunctional immune response [12, 13]. The fact that T regulatory (Treg) and CD4^+^ helper T (Th) cells (Th1, Th2, Th17 cells) are crucial for the development of HSP and HSPN supports this hypothesis [14].

RETRACTED

In a healthy human, the gut microbiome is a complex community of over 100 trillion microbes, representing more than 1,000 species [15] and encoding 3.3 million genes, a number that is 100-fold greater than the number of human genes [16]. Major phyla in gut microbiota include *Bacteroides*, *Firmicutes*, *Actinobacteria*, and *Proteobacteria* [17]; their compositions and metabolites are important for critical immune processes, such as shaping B cell repertoires, antibody production, Th17 cell subpopulation regulation, Th17/Treg balance maintenance, and controlling Th subpopulation homeostasis [17, 18]. Changes in the gut microbiome are being increasingly linked to various disorders, including inflammatory bowel disease, cancer, obesity, diabetes, cardiovascular disease, and kidney disease [19, 20].

In this study, we aimed to differentiate between HSP and HSPN through an analysis of gut microbiome composition, using fecal samples from children with the two conditions. We hope to provide data that would enable the development of new therapeutic approaches for HSP and HSPN.

RETRACTED

## 2. Methods

### 2.1. Study Cohort

Children with HSP (Group A, *n* =25) were recruited from Hangzhou Children's Hospital and The Children's Hospital of Zhejiang University School of Medicine, Hangzhou, China. All children were diagnosed with HSP based on the 2010 EULAR/PRINTO/PReS criteria for the classification of childhood vasculitis [21]. Children with HSPN (Group B, *n* =25) were recruited from Hangzhou Children's Hospital and The Children's Hospital of Zhejiang University School of Medicine, Hangzhou, China. All children with HSPN showed symptoms corresponding to the criteria used for diagnosing this condition [22]. Finally, 25 healthy children (Group C) were recruited as controls from Hangzhou Children's Hospital. Patients with concomitant diseases or a history of gastrointestinal surgery were excluded from the analysis. None of the subjects received antibiotics, probiotics, corticosteroids, or immunosuppressants for 3 months before fecal collection. All fecal samples were transported in liquid nitrogen and stored at −80°C until bacterial DNA extraction. Ethical approval was obtained from the Ethics Committee of Hangzhou Children's Hospital.

### 2.2. DNA Extraction and Amplification of V3-V4 Regions

Total bacterial DNA was extracted from fecal samples using a QIAamp DNA Stool Mini Kit (Qiagen, Duesseldorf, Germany) following the manufacturer's protocol. Illumina (San Diego, CA, USA) overhang adapter sequences were added to gene-specific sequences. The following full-length primers were used to target the V3-V4 of the *16S rRNA* gene: forward, 5′ TCGTCGGCAGCGTCAGATGTGTATAAGAGACAGCCTACGGGNGGCWGCAG 3′ and reverse 5′ GTCTCGTGGGCTCGGAGATGTGTATAAGAGACAGGACTACHVGGGTATCTAATCC 3′.

### 2.3. MiSeq Sequencing

High-throughput sequencing of the *16S rRNA* gene was performed by G-Bio (Hangzhou, China) using MiSeq (Illumina, San Diego, CA, USA). The ends of paired 300 bp reads were overlapped using MiSeq v3 reagents to generate high-quality, full-length reads of the V3 and V4 regions in a single 65 h run. Products were normalized at equimolar concentrations and subjected to paired-end sequencing (2 × 300 cycles) on the MiSeq Benchtop Sequencer, following standard protocols.

### 2.4. Quantitative Analysis of 16S rRNA Genes, Operational Taxonomic Unit (OTU) Clustering, and Rarefaction Curve

Quantitative PCR (qPCR) was validated by constructing an artificial mixture of *16S rRNA* genes following established protocols. After sample loading, the metagenomic workflow built into the MiSeq Reporter was used to perform taxonomic analysis using 16S rRNA data from the Greengenes database (http://greengenes.lbl.gov/). The output of this workflow was a classification of reads at all taxonomic levels (kingdom, phylum, class, order, family, genus, and species). However, only genera and species were graphically depicted.

RETRACTED

### 2.5. Bioinformatics Analysis

Raw, paired reads were checked with QIIME quality filters under the default settings for Illumina processing. Clean reads were chimera-checked with the gold.fa database (http://drive5.com/uchime/gold.fa) and clustered into OTUs (97% similarity cutoff) with the Search pipeline. The OTUs were classified based on Ribosomal Database Project (RDP) Release 9.201.203. Alpha diversity using Chao1 was determined in RDP-classifier. Bray–Curtis dissimilarity was calculated to determine beta diversity.

### 2.6. Statistical Methods

Principal coordinate analysis (PCoA), principal component analysis (PCA), and analysis of similarities (ANOSIM) were all performed using R (Vegan package, V3.3.1). The former two analyses determined differences in OTU relative abundance between groups, whereas the latter determined differences in microbial community composition. All other analyses were performed using SPSS version 22.0. Data are presented as means ± SD. Significance was set at *p* < 0.05.

## 3. Results

### 3.1. Clinical Characteristics

The age of onset was 6.7 ± 2.2 years among children with HSP (boys: girls, 13 : 12). Among children with HSPN (boys: girls, 15 : 10), the age of onset was 8.7 ± 2.7 years. The average age of the healthy controls (boys: girls, 14 : 11) was 6.0 ± 2.2 years. The most common clinical characteristics of HSP include skin purpura, joint involvement, abdominal pain, vomiting, and/or gastrointestinal hemorrhage. HSPN presents with significant clinical manifestations, including microalbuminuria to massive proteinuria, microscopic hematuria to gross hematuria, proteinuria and hematuria, and acute renal insufficiency (ARI) (Table 1).

### 3.2. Gut Microbiota Variation

Gut microbial richness was evaluated using Chao1 and the number of OTUs. Rarefaction curves showed that the diversity of gut microbiota differed significantly between children with HSP and children with HSPN. At the same time, represented data demonstrated no significant difference between HSP children and healthy children (Figure 1; *P* = 0.0224).

The top five most abundant microbial genera were *Bacteroides*, *Faecalibacterium*, *Prevotella*, *Ruminococcaceae*, and *Megamonas* in children with HSP; *Bacteroides*, *Faecalibacterium*, *Prevotella*, *Bifidobacterium*, and *Ruminococcaceae* in children with HSPN; *Bacteroides*, *Prevotella*, *Faecalibacterium*, *Ruminococcaceae*, and *Bifidobacterium* in healthy controls (Figure 2).

*Bifidobacterium* abundance was the lowest among children with HSP (Figure 3; *P* < 0.05). Children with HSPN had a lower *Akkermansia* abundance than that of children with HSP (Figure 3; *P* < 0.05). Children with HSPN also had a markedly higher *Alistipes* abundance than that of the other two groups (Figure 3; *P* < 0.05).

RETRACTED

The structure of intestinal microbiota was similar across all three groups, according to PCA and PCoA (Figure 4). Additionally, we found no intra-group differences in the composition of fecal microbial communities (Figure 5; ANOSIM, *R* = −0.002, *P* = 0.46).

## 4. Discussion

In this study, we successfully examined how HSP and HSPN altered the gut microbiota of children in China, demonstrating that the two diseases were associated with dysbiosis. However, the composition of gut microbiota did not significantly differ between children with HSP, children with HSPN, and healthy children. At the same time, represented data demonstrated that the diversity of gut microbiota was not significantly different between HSP children and healthy children. This is not consistent with literature reports [23].

Gut microbiota is crucial for the health and influences susceptibility to disease [24], specifically by modulating immune responses [25, 26]. Here, we observed that *Bifidobacterium* abundance was lower among children with HSP than in children with HSPN. *Bifidobacterium* is a common probiotic due to its ability to suppress inflammation and improve epithelial cell barrier resistance [27]. In children with HSP, *Bacteroides* and *Lachnoclostridium* may influence IgG and complement C3 levels. The gut microbiome was linked to abdominal complaints in HSP children (Streptococcus and butyric acid-producing bacteria). Previous research has suggested that members of this genus can restore intestinal permeability, cytokine levels in different barrier injury models, and colonic goblet cell populations [28, 29]. Another study found that *Bifidobacterium* was less abundant in the guts of patients with HSP than in the guts of healthy controls, but this difference was not significant [23].

Another key difference between children with HSP and those with HSPN was that the latter exhibited a lower *Akkermansia* abundance. Mucin-degrading bacteria *Akkermansia* is widely found in the human stomach. These results correspond with those of studies demonstrating that *Akkermansia* abundance decreases markedly in patients with chronic kidney disease and is negatively correlated with IL-10 levels [30]. *Akkermansia* comprises 1–4% of total gut microbiota; its known functions include providing energy to the host, degrading mucin, and producing short-chain fatty acids and propionic acids [31]. *Akkermansia* abundance in the gut is negatively correlated with obesity, diabetes, and appendicitis [32]. Furthermore, patients with HSPN also had the highest relative *Alistipes* abundance, which was previously shown to rise concurrently with an increase in DNA damage-causing bacteria [33].

RETRACTED

In this study, we showed that the gut microbiota of children with HSP and HSPN exhibited clear dysbiosis. Children with HSP had the lowest *Bifidobacterium* abundance, while children with HSPN had lower *Akkermansia* abundance than children with HSP did. Furthermore, *Alistipes* was the most abundant genus in children with HSPN.

The study was very preliminary. It was not clear the relationship between the International Study of Kidney Disease in Children (ISKDC) grading and gut microbiota. The small sample size limited the applicability of our study to a wider population. Further studies should therefore aim to perform investigations using a larger sample size. Nevertheless, our findings provide important insights for the development of microbe-based therapies that can improve the clinical outcomes of HSP and HSPN and even prevent their development. Given the findings of dysbiosis, we recommend performing evaluations as to how probiotic supplementation may influence the treatment of HSP or HSPN in children.

## Figures and Tables

**Figure 1:** Diversity analysis of *16S rRNA* gene sequences obtained from fecal samples of groups A (children with Henoch-Schonlein purpura), B (children with Henoch-Schonlein purpura nephritis), and C (healthy controls).

**Figure 2:** Composition of microbial genera. Composition of fecal microbiota in groups A, B, and C at the genus level. The relative abundance of microbial genera was determined. Each column represents one fecal sample, and the ordinate indicates the relative abundance.

**Figure 3:** Relative abundance of bacterial genera. The abundance and diversity of the top 20 bacterial genera were compared across groups A, B, and C. Red font indicates significant differences (*P* < 0.05).

**Figure 4:** PCA and PCoA distance function. Visualization of PCA and PCoA results for fecal samples from groups A, B, and C.

**Figure 5:** Dissimilarity rank distribution. Comparison of the gut microbial community composition between groups A, B, and C using analysis of similarities (ANOSIM).

**Table 1:** Clinical manifestations of HSP and HSPN.

Group	Skin purpura (*n*)	Joint involvement (*n*)	Abdominal pain and/or vomiting (*n*)	Gastrointestinal hemorrhage (*n*)	Hematuria (*n*)	Proteinuria (*n*)	Hematuria and proteinuria (*n*)	ARI (*n*)
Group A (HSP)	24	12	11	4	0	0	0	0
Group B (HSPN)	25	12	14	6	8	13	4	0

## Data Availability

The data used to support the findings of this study are available from the corresponding author upon request.
